RETRACTED

# RNAi targeting CXCR4 inhibits proliferation and invasion of esophageal carcinoma cells

**DOI:** 10.1186/1746-1596-8-104

**Published:** 2013-06-24

**Authors:** Tao Wang, Yanfang Mi, Linping Pian, Ping Gao, Hong Xu, Yuling Zheng, Xiaoyan Xuan

**Affiliations:** 1 Department of Hemato-tumor, The First Affiliated Hospital of Henan College, University of TCM, Zhengzhou, P.R. China; 2 The First Affiliated Hospital of Zhengzhou University, Zhengzhou 450052, P.R. China; 3 Department of Otolaryngology Head and Neck Surgery, The Second Affiliated Hospital of Zhengzhou University, Zhengzhou P.R. China; 4 Department of Ultrasound, The First Affiliated Hospital College, TCM of Henan, Zhengzhou P.R. China; 5 Henan Tumor Institute, Zhengzhou, P.R. China; 6 Henan University of TCM, Zhengzhou, P.R. China; 7 College of Basic Medical Sciences, Zhengzhou University, Zhengzhou, P.R. China

**Keywords:** Esophageal carcinoma, CXCR4, Proliferation, Invasion

## Abstract

CXC chemokine receptor 4 was found to be expressed by many different types of human cancers and its expression has been correlated with tumor aggressiveness, poor prognosis and resistance to chemotherapy. However the effect of CXCR4 on the esophageal carcinoma cells remains unclear, the present study explored the effects of CXCR4 siRNA on proliferation and invasion of esophageal carcinoma KYSE-150 and TE-13 cells. Two siRNA sequence targeting CXCR4 gene were constructed and then were transfected into KYSE-150 and TE-13 cells by Lipofectamine™2000. Changes of CXCR4 mRNA and protein were analyzed by qRT-PCR and Western blot. Effect of CXCR4 siRNA on KYSE-150 and TE-13 cells proliferation was determined by MTT. Transwell invasion assay was used to evaluate the invasion and metastasis of KYSE-150 and TE-13 cells. Tumor growth was assessed by subcutaneous inoculation of cells into BALB/c nude mice. qRT-PCR and Western blot demonstrate that the expression level of CXCR4 gene were obviously decreased in KYSE-150 and TE-13 cells transfected with CXCR4 targeting siRNA expression vectors. The average amount of cells transfected with CXCR4 siRNA penetrating Matrigel was significantly decreased (p<0.05). Injection of CXCR4 siRNA transfected cells inhibited tumor growth in a xenograft model compared with blank and negative control groups (p <0.05). CXCR4 silenced by siRNA could suppress the proliferation, invasion and metastasis of esophageal carcinoma cell lines KYSE-150 and TE-13 in vitro and in vivo. The results provide a theoretical and experimental basis for the gene therapy of ESCC using RNAi technology based on CXCR4 target site.

**Virtual slides:**

The virtual slide(s) for this article can be found here: http://www.diagnosticpathology.diagnomx.eu/vs/3502376691001138

RETRACTED

## Introduction

ESCC is one of the most common malignant tumors in China, and the early invasion is the main reason for its poor prognosis [1-3]. In recent years, the role of chemokine receptor in cancer cell invasion and metastasis have been concerned widely all over the world. CXCR4 (CXC chemokine receptor 4, CXCR4) is a receptor of SDF-1 (stromal cell – derived factor-1, SDF-1). CXCR4 was found to be expressed in many different types of human cancers and its expression has been correlated with tumor aggressiveness, poor prognosis and resistance to chemotherapy [4-6]. These findings suggest that CXCR4 is a potentially attractive therapeutic target. However the effect of CXCR4 on the esophageal carcinoma cells remains unclear, the present study examined the effect of CXCR4 on the proliferation and invasion of the esophageal carcinoma cell lines KYSE-150 and TE-13.

## Materials and methods

### Cells and cell culture

The human esophageal carcinoma cell line KYSE-150 and TE-13 were purchased from the Chinese Academy of Sciences Cell Bank. All cells were cultured in RPMI-1640 (Gibco, USA) supplemented with 10% fetal bovine serum (Invitrogen, Carlsbad, USA) and grown in a 37°C, 5% CO_2_ incubator.

### Oligonucleotides and cell transfection

The oligonucleotides used in this study were chemically synthesized by Sangon Co. Ltd (Shanghai, China). The sequences used were as follows: siRNA1: sense, 5'-UAAAAUCUUCCUGCCCACCdTdT-3', siRNA2: sense, 5'-GGAAGCUGUUGGCUGAAAAdTdT-3' Negative control siRNA: sense, 5′ GGUGAACUGUCUGGAUAAG 3′.For transfection, 2×10^5^ cells were seeded into each well of six well plates and grown overnight until they were 50–80% confluent. Cells were washed, placed in serum-free medium and transfected with siRNA using Lipofectamine™2000 according to the manufacturer’s instructions (Invitrogen). After 6 h, the medium was changed to complete medium, and cells were cultured at 37°C in 5% CO_2_. Four groups were generated for all experiments, a blank control group (blank control); a negative control group (negative control); and a siRNA1 group (siRNA1); a siRNA2 group (siRNA2).

### Real time PCR analysis

Total RNA was extracted using the Trizol Reagent (Invitrogen, USA) according to the manufacturer’s instructions. Reverse transcription and amplification were performed using a qPCR Quantitation Kit. The ABI 7300 HT Sequence Detection system (Applied Biosystems, Foster City, CA, USA) was used to detect the relative levels of CXCR4 in siRNA-transfected cells. The amplification reaction (40 μl) included 2× real-time Buffer (20 μl), the special primer set (0.8 μl), ddH2O (18 μl), cDNA (1 μl), and 5 U/μl Taq DNA polymerase (0.2 μl).

RETRACTED

For CXCR4 (470 bp), forward: 5'-ACCGAGGAAATGGGCTCAGGG-3'; reverse: 5'-ATAGTCAGCAGGAGGGCAGGGA -3'. The reaction conditions were as follows: stage 1, 95°C for 3 min (1 cycle); stage 2, 95°C for 14 s followed by 65°C for 45 s (40 cycles); stage 3, from 62°C up to 95°C followed by 0.2°C for 2 s (1 cycle). The results of real-time PCR were analyzed by the DDCt method. Quantitative CXCR4 expression data were calculated using 2^-Ct^. The experiments were performed independently four times.

### Western blot analysis

The four experimental groups of cells were lysed for total protein extraction. The protein concentration was determined by the BCA method (KeyGEN, China), and 30 μg of protein lysates were subjected to SDS-PAGE. The electrophoreses proteins were transferred to nitrocellulose membranes (Whatman, USA), which were blocked in 5% non-fat milk and incubated overnight at 4°C with diluted antibodies against CXCR4 (1:800, Cell Signaling Technology, USA), Membranes were then incubated with HRP-conjugated secondary antibody (1:2,500, Santa Cruz, USA). After washing with PBST buffer (PBS containing 0.05% Tween-20), membranes were probed using ultra-enhanced chemiluminescence western blotting detection reagents. GAPDH was used as the internal reference. The experiments were performed independently four times.

### Transwell invasion assay

Transwell filters (Costar, USA) were coated with matrigel (3.9 μg/μl, 60–80 μl) on the upper surface of the polycarbonic membrane (6.5 mm in diameter, 8 μm pore size). After 30 min of incubation at 37°C, the matrigel solidified and served as the extracellular matrix for tumor cell invasion analysis. Cells were harvested in 100 μl of serum free RPMI-1640 medium and added to the upper compartment of the chamber. The cells that had migrated from the matrigel into the pores of the inserted filter were fixed with 100% methanol, stained with hematoxylin, mounted, and dried at 80°C for 30 min. The number of cells invading the matrigel was counted from three randomly selected visual fields, each from the central and peripheral portion of the filter, using an inverted microscope at 200× magnification. The experiments were performed independently four times.

### MTT assay

Cell proliferation was assessed by the MTT (Moto-nuclear cell direc cytotoxicityassay) [3-(4,5-dimethylthiazol-2-yl)-2,5-diphenyltetrazoliumbromide]assay. The four experimental groups of cells were plated at 1 × 10^3^ cells/well on 96-well plates. 20 μL of MTT (5 mg/mL) was added to each well after 48 h and then sub-cultured in the medium with 100 μL DMSO. The absorbance of each well was determined at 490 nm. The experiments were performed independently four times.

RETRACTED

### Nude mouse tumor xenograft model

Forty immunodeficient female BALB/C nude mice, 5–6 weeks old (purchased from the Experimental Animal Center of the Henan province, China) were randomly divided into eight groups (four groups per cell line, five mice per group). They were bred under aseptic conditions and maintained at constant humidity and temperature. This study was carried out in strict accordance with the recommendations in the Guide for the Care and Use of Laboratory Animals of Zhengzhou University. The protocol was approved by the Committee on the Ethics of Animal Experiments of Zhengzhou University. All surgery was performed under sodium pentobarbital anesthesia, and all efforts were made to minimize suffering. Mice in the different groups were subcutaneously injected in the dorsal scapular region with the corresponding cells from each experimental condition. Tumors were harvested after four weeks.

### Nude mouse tumor xenograft immunohistochemical analysis

Select the four groups of tumor tissue respectively, formalin-fixed, paraffin-embedded specimens and tissue sections. HE staining observed the pathological changes of the tumor under a microscope. Observe the expression of CXCR4 protein with the method of immunohistochemical SP staining. The positive color is brown particles. Each film were counted 5 high power field (400 x), each of the visual observation of 200 cells and recording the value of the positive cells as a result of statistical analysis, calculate the average number of positive cells in the cells of each array was 200. No coloration is negative.

### Statistical analysis

SPSS17.0 was used for statistical analysis. One-way analysis of variance (ANOVA) and the χ2 test were used to analyze the significance between groups. Multiple comparisons between the parental and control vector groups were made using the Least Significant Difference test when the probability for ANOVA was statistically significant. All data represent mean±SD. Statistical significance was set at p<0.05.

## Results

### CXCR4 siRNA inhibited significantly the mRNA expression of CXCR4

After siRNA interference KYSE-150 for 48 h, compared with negative control and blank control group, CXCR4 mRNA expression was inhibited in CXCR4 siRNA1 group and CXCR4 siRNA2 group. TE-13 cells using the targeting CXCR4 siRNA interference after 48 h, RT-PCR results also showed that CXCR4 mRNA expression in CXCR4 siRNA1 group and siRNA2 group was inhibited compared to negative control and blank control group as shown in Figure 1, the targeted CXCR4 siRNA inhibited significantly the mRNA expression of CXCR4 gene.

**Figure 1:** **CXCR4 siRNA inhibited significantly the mRNA expression of CXCR4.** Cells were incubated with different synthetic oligonucleotides as described in the materials and methods section, and CXCR4 mRNA was quantified by real time PCR. The targeted CXCR4 siRNA inhibited significantly the expression of CXCR4 gene (*p <0.05).

RETRACTED

### CXCR4 siRNA inhibited significantly the protein expression of CXCR4

After siRNA1 and siRNA interference KYSE-150 for 48 h, Western-Blot results showed that CXCR4 protein was decreased by 50.6% and 45.6% respectively, compared with negative control group. TE-13 cells using siRNA1 and siRNA interference after 48h, Western-Blot results also showed that CXCR4 protein was decreased by 54.1% and 44.4% compared with negative control group (Figure 2). The results showed that CXCR4 siRNA1 and siRNA2 not only effectively inhibit the expression of CXCR4 mRNA, but also play an effective inhibition for CXCR4 protein expression, and targeting CXCR4 siRNA1 interference effect is more obvious.

**Figure 2:** **CXCR4 siRNA inhibited significantly the protein expression of CXCR4.** Cells were incubated with different synthetic oligonucleotides as described in the materials and methods section, and CXCR4 protein was quantified by Western-Blot. The targeted CXCR4 siRNA inhibited significantly the protein expression of CXCR4 gene (*p <0.05).

### siRNA CXCR4 reduced esophageal carcinoma cells invasion in vitro

In order to detect the effects of CXCR4 on invasion of esophageal carcinoma, we used transwell invasion assay and found that KYSE-150 and TE-13 penetrating cells transfected with CXCR4 siRNA1 and CXCR4 siRNA2 reduced significantly compared to negative control and blank control group (Figure 3). It is no significant difference between negative control and blank control group. siRNA CXCR4 gene significantly inhibited esophageal squamous cell carcinoma KYSE-150 and TE-13 cells invasion ability in vitro.

**Figure 3:** **siRNA CXCR4 reduced esophageal carcinoma cells invasion in vitro.** Cells were incubated with different synthetic oligonucleotides as described in the materials and methods section, and cells invasion ability was deteced by transwell invasion assay. The targeted CXCR4 siRNA reduced esophageal carcinoma cells invasion ability (*p <0.05).

### siRNA CXCR4 inhibited esophageal carcinoma cells proliferation in vitro

In order to explore the effects of CXCR4 on proliferation of esophageal carcinoma, we used MTT experiment. The results showed that absorbance value (A value) of KYSE-150 and TE-13 cells transfected with the CXCR4 siRNA1 and CXCR4 siRNA2 decreased significantly (Figure 4). It can be seen that inhibition of CXCR4 expression in vitro could not only decreased the invasion and metastasis but also inhibit the proliferation.

RETRACTED

**Figure 4:** **siRNA CXCR4 inhibited esophageal carcinoma cells proliferation in vitro. A**. TE-13 cells were incubated with different synthetic oligonucleotides as described in the materials and methods section, and cells proliferation was detected by MTT assay. The targeted CXCR4 siRNA inhibited esophageal carcinoma TE-13 cell proliferation. **B**. KYSE-150 cells were incubated with different synthetic oligonucleotides as described in the materials and methods section, and cells proliferation was detected by MTT assay. The targeted CXCR4 siRNA inhibited esophageal carcinoma KYSE-150 cell proliferation.

### The growth inhibitory effects of CXCR4 were examined in vivo using a xenograft model of esophageal cancer

Nude mice were inoculated KYSE-150 and TE-13 cells after about one week, all nude mice have tumor, inoculation site appears small subcutaneous nodules. At first, tumor was oval, later becoming irregular, uneven surface. After the mice died four weeks later, strip nude mice tumor and weigh by electronic balance. The results showed that tumor weight of CXCR4 siRNA1 and CXCR4 siRNA2 group was significantly lower than that negative control and blank control group in the nude mouse, the difference have a statistically significant (p <0.05) (Figure 5). There was no significant difference (p > 0.05) of tumor weight between negative control and blank control group. The results showed that the siRNA of targeting CXCR4 inhibited tumor growth in a xenograft model.

**Figure 5:** **The growth inhibitory effects of CXCR4 were examined in vivo using a xenograft model of esophageal cancer. A**. Nude mice were inoculated KYSE-150. Four weeks later, strip nude mice tumor and weigh by electronic balance. The targeted CXCR4 siRNA inhibited tumor growth in a xenograft model (*p <0.05). **B**. Nude mice were inoculated TE-13 cells. Four weeks later, strip nude mice tumor and weigh by electronic balance. The targeted CXCR4 siRNA inhibited tumor growth in a xenograft model.

### CXCR4 siRNA inhibited xenografts tumor tissue CXCR4 mRNA expression effectively in vivo

In nude mice esophageal carcinoma cell xenografts model, expression of CXCR4 mRNA in CXCR4 siRNA1 and CXCR4 siRNA2 group were lower significantly than in negative control and blank control group (Figure 6), The results showed that CXCR4 siRNA inhibited xenografts tumor tissue CXCR4 mRNA expression effectively in vivo.

**Figure 6:** **CXCR4 siRNA inhibited xenografts tumor tissue CXCR4 mRNA expression effectively in vivo.** In nude mice esophageal carcinoma cell xenografts model, xenografts tumor tissue CXCR4 mRNA expression was quantified by real time PCR. CXCR4 siRNA inhibited xenografts tumor tissue CXCR4 mRNA expression in vivo (*p <0.05).

RETRACTED

### The histopathologic changes of nude mice tumor tissues

The histopathologic changes of tumor tissues from two nude mice models bearing esophageal carcinoma were observed using HE stains. The tumor cells in group CXCR4 siRNA1 and CXCR4 siRNA2 had apoptosis and necrosis. Morphology was different from each other, furthermore, nuclei showed pathological division and the giant tumor cells were rare (Figure 7). While the tumor cells in negative control and blank control group were sheet arranged, size were different from each other, nuclei were large and showed multi morphology, pathological cell division and giant tumor cells were in much with marked atypia.

**Figure 7:** **The histopathologic changes of nude mice tumor tissues.** The histopathologic changes of tumor tissues from two nude mice models bearing esophageal carcinoma were observed using HE stains. The tumor cells in group CXCR4 siRNA1 and CXCR4 siRNA2 had apoptosis and necrosis, morphology was different from each other, nuclei showed pathological division and the giant tumor cells were rare (400 x).

### CXCR4 protein expression of CXCR4 siRNA1 group was reduced in nude mice xenografts

Compared with negative control and blank control group, CXCR4 protein expression of CXCR4 siRNA1 and CXCR4 siRNA2 group was significantly reduced in the two types of esophageal cell xenografts model in nude mice, the difference was significant (p <0.05)(Table 1 and Figure 8).

**Figure 8:** **CXCR4 siRNA inhibited significant CXCR4 protein expression.** The expression of CXCR4 protein was observed with the immunohistochemical SP staining. The positive color is brown particles. CXCR4 siRNA inhibited significant CXCR4 protein expression.

**Table 1:** The positive expression number of CXCR4 protein in nude mice xenografts

**Groups**	**n**	**KYSE-150 nude mice**	**TE-13 nude mice**
CXCR4siRNA1	200	81±5^*^	86±5^*^
CXCR4siRNA2	200	97±4^*^	92±6^*^
negative control	200	140±8	132±7
blank control	200	143±4	148±3

The positive color is brown particles. Each film were counted 5 high power field (400 x), each of the visual observation of 200 cells and recording the value of the positive cells as a result of statistical analysis, calculate the average number of positive cells in the cells of each array was 200. No coloration is negative. Compared with negative control and blank control group, CXCR4 protein expression of CXCR4 siRNA1 and CXCR4 siRNA2 group was significantly reduced in the two types of esophageal cell xenografts model in nude mice, the difference was significant (* p <0.05).

RETRACTED

## Discussion

Chemokine receptors are parts of G protein-coupled receptor superfamily whose function is changing by cell types and activities. A large amount of chemokine and receptor reactions are produced by the different combination of ligand and receptor. CXCR4 is a 7-transmembrane G-coupled receptor which belongs to the chemokine receptors family, and is expressed by variety of cells during development and adult life. Its unique ligand is SDF-1, CXCL12 in systematic name. SDF-1 and CTCR4 have a high affinity and their specific binding, SDF-1–CXCR4 axis, is the molecular basis of the biological function which plays an important role in cell communication and cell migration [4,5]. Chemokine receptor, CXCR4, was first reported high expression in human breast tumor and its’ metastasis by Mullar A etc. [7]. In breast cancer cell, polymerization of reactive protein and formation of pseudopod were mediated by CXCR4 signal transduction pathway who leads chemotaxis and invade reactions latter [8]. As the research of CXCR4 gene continues, 23 kinds of cancer cells, at least, until now, were found that have selective high expression about it, including ovarian cancer, renal cell carcinoma, colorectal cancer, melanoma, esophageal cancer and so on [9-23].

Nowadays, RNAi has become a powerful strategy for knockdown and for understanding gene function. RNAi is a general mechanism for the sequence-specific gene-silencing induced by double stranded RNA [24]. RNAi, mediated by small interfering RNA (siRNA), is a double stranded form of RNA that is about 21–23 nucleotide long and is specific for the sequence of its target [25]. For siRNA to be a useful tool in gene knockdown experiments and ultimately for therapeutic purposes, siRNA-mediated transcriptional silencing must be specific. Many studies [26-30] have shown that siRNA mediated gene silencing can be a reliable and valuable approach for large-scale screening of gene function and drug-target identification and validation.

Esophageal cancer is one of the most common malignant tumors in China. Though the diagnosis and treatment of esophageal carcinoma have developed much these years, the esophageal carcinoma runs quickly in clinical and has a worse prognosis for its invasion and metastasis in the early stage [31,32]. For the further study about the effect of SDF-1–CXCR4 axis on the invasion and metastasis of ESCC and provide the new target spot to remedy ESCC, the siRNA for CXCR4 were designed to research the effects of CXCR4 on proliferation and invasion of esophageal carcinoma. Two siRNA vectors aiming to CXCR4 gene were constructed. CXCR4 siRNA was transfected into KYSE-150 and TE-13 cells by Lipofectamine™2000. Changes of CXCR4 mRNA and protein were analyzed by RT-PCR and Western blot. The results showed that the two siRNA sequence target gene of CXCR4 could both restrain the expression of ECSS CXCR4 gene and the interference effect of siRNA 1 was better. It means that different target sites make different interference effects. The transwell results indicated that the numbers of penetrating cells transfected with CXCR4 siRNA1 and CXCR4 siRNA2 reduced significantly compared to negative control and blank control group, which showed CXCR4 silenced by siRNA could suppress the proliferation, invasion and metastasis of esophageal carcinoma cell lines KYSE-150 and TE-13.

RETRACTED

For the purpose of verifying the function of CXCR4 siRNA in vivo, the animal model of xenograft tumor of carcinoma of esophagus was structured using KYSE-150 and TE-13. In the xenograft tumor, it showed that tumors of the CXCR4 siRNA group were restrained obviously. The further experiment indicated that the CXCR4 mRNA and the protein expression were obviously lower than the control groups, and the tumor cells had apoptosis and necrosis. Morphology were different from each other, furthermore, nuclei showed pathological division and the giant tumor cells were rare. CXCR4 siRNA could not only, in vivo, interfere with CXCR4 gene and affect cell proliferation of KYSE-150 and TE-13 cell, but also decrease the expression of CXCR4 and suppress tumor growth in vivo. The results provide a theoretical and experimental basis for the gene therapy of ESCC using RNAi technology based on CXCR4 target site.

## Conclusions

CXCR4 silenced by siRNA could suppress the proliferation, invasion and metastasis of esophageal carcinoma cell lines KYSE-150 and TE-13 in vitro and in vivo. The results provide a theoretical and experimental basis for the gene therapy of ESCC using RNAi technology based on CXCR4 target site.

## Competing interests

The authors declare that they have no competing interests.

## Authors’ contributions

XYX, LPP and TW: conceived of the study, and participated in its design and coordination and helped to draft the manuscript. PG, HX and YLZ: carried out part of experiments and wrote the manuscript. LPP and TW performed the statistical analysis. All authors read and approved the final manuscript.
